# Liraglutide inhibits autophagy and apoptosis induced by high glucose through GLP-1R in renal tubular epithelial cells

**DOI:** 10.3892/ijmm.2014.2052

**Published:** 2014-12-29

**Authors:** X ZHAO, G LIU, H SHEN, B GAO, X LI, J FU, J ZHOU, Q JI

**Affiliations:** Department of Endocrinology, The First Affiliated Hospital of The Fourth Military Medical University, Xi’an, Shaanxi, P.R. China

**Keywords:** high glucose, autophagy, autophagy-related gene, glucagon-like peptide-1 receptor, liraglutide

## Abstract

Tubular atrophy and dysfunction is a critical process underlying diabetic nephropathy (DN). Understanding the mechanisms underlying renal tubular epithelial cell survival is important for the prevention of kidney failure associated with glucotoxicity. Autophagy is a cellular pathway involved in protein and organelle degradation. It is associated with many types of cellular homeostasis and human diseases. To date, little is known of the association between high concentrations of glucose and autophagy in renal tubular cells. In the present study, we investigated high glucose-induced toxicity in renal tubular epithelial cells by means of several complementary assays, including cell viability, cell death assays and changes in ultrastructure in an immortalized human kidney cell line, HK-2 cells. The extent of apoptosis was significantly increased in the HK-2 cells following treatment with high levels of glucose. In addition, in *in vivo* experiments using diabetic rats, high glucose exerted harmful effects on the tissue structure of the kidneys in the diabetic rats. Chronic exposure of the HK-2 cells and tubular epithelial cells of nephritic rats to high levels of glucose induced autophagy. Liraglutide inhibited these effects; however, treatment witht a glucagon-like peptide-1 receptor (GLP-1R) antagonist enhanced these effects. Our results also indicated that the exposure of the renal tubular epithelial cells to high glucose concentrations *in vitro* led to the downregulation of GLP-1R expression. Liraglutide reversed this effect, while the GLP-1R antagonist promoted it, promoting autophagy, suggesting that liraglutide exerts a renoprotective effect in the presence of high glucose, at least in part, by inhibiting autophagy and increasing GLP-1R expression in the HK-2 cells and kidneys of diabetic rats.

## Introduction

The number of patients with diabetes is markedly increasing worldwide. Diabetes leads to vascular changes and dysfunction, as well as complications that result in increased morbidity and mortality (1). Among diabetic vascular complications, nephropathy contributes to the development of cardiovascular disease and is the leading cause of end-stage renal disease in developed countries (2,3). Therefore, the prevention of renal insufficiency may improve the prognosis of patients with diabetes.

Numerous factors contribute to the development of diabetic nephropathy. Hyperglycemia alters both extracellular and intracellular metabolism, leading to effects such as glomerular hyperfiltration (4), oxidative stress (5), the accumulation of advanced glycation end products (AGEs) (6), the activation of protein kinase C (7), abnormal polyol metabolism (8), the overexpression of transforming growth factor-β (TGF-β) (9) and inflammation. These effects have been recognized as classical characteristics of the pathogenesis of diabetic nephropathy. Additionally, intracellular stress associated with renal hypoxia (10,11), reactive oxygen species (ROS) production by mitochondria (12–15) and endoplasmic reticulum (ER) stress (16–18) have recently been proposed as key mechanisms underlying the pathogenesis of diabetic nephropathy. Thus, the maintenance of cellular homeostasis against stress conditions may be a new therapeutic target for the treatment of diabetic nephropathy.

Autophagy is a tightly regulated process in which endogenous cellular proteins aggregate and damaged organelles are degraded by the lysosomal pathway. This process functions to maintain intracellular homeostasis and cell integrity. It has recently been highlighted as it can be stimulated by multiple types of cellular stressors, including starvation, hypoxia and ER stress. Emerging evidence also indicates that autophagy plays a critical role in several organs, particularly in highly metabolic organs, and that its alteration is involved in the pathogenesis of metabolic disease, immunity and autoimmunity, inflammation, development, aging and cancer (19,20). It has been suggested that autophagy is enhanced and plays a protective role during kidney disease (21). Its renoprotective role in several animal models, including those used for aging and acute kidney injury, has also been demonstrated (22–24).

One possible mechanism through which autophagy protects cells is that it may eliminate damaged mitochondria. Autophagy involves the sequestration of proteins and cellular organelles into autophagosomes, which directs them to lysosomes (25). The formation of autophagosomes is dependent on the induction of several genes, including microtubule-associated protein 1 light chain 3 (LC3), Beclin1 and autophagy-related genes (Atgs) (26). Nonetheless, autophagy may also represent a form of programmed cell death known as autophagic cell death or type II programmed cell death, and altered autophagy is associated with the loss of renal tubular epithelial cell mass in diabetes. The role of autophagy in diabetic nephropathy remains a largely undetermined; thus, its underlying mechanisms are presently unclear.

Glucagon-like peptide-1 (GLP-1) is a gut incretin hormone and is currently considered an attractive agent for the treatment of type 2 diabetes. It has been shown to exert various beneficial effects on pancreatic β-cells, such as the enhancement of glucose-dependent insulin secretion (27), the acceleration of β-cell proliferation and the inhibition of β-cell apoptosis (28). In the gut and hypothalamus, GLP-1 has been shown to inhibit motility, gastric emptying (29) and the central regulation of feeding (30), resulting in the loss of body weight (27). It has previously been demonstrated that GLP-1 receptor (GLP-1R) is produced not only in the pancreas, gut and hypothalamus, but also in the kidneys (31). Liraglutide is a human incretin-GLP-1 analogue with a high degree of homology to the native hormone. It shares 97% sequence identity with native human GLP-1. A recent study demonstrated that liraglutide inhibited cytokine-induced apoptosis in primary rat islet cells in a dose-dependent manner and reduced free fatty acid-induced apoptosis by approximately 50% (32).

In the present study, we evaluated the effects of high glucose concentrations on the induction of autophagy in the human renal tubular epithelial cell line, HK-2 cells, as well as in the kidneys of diabetic rats. We also investigated the ability of GLP-1 to protect HK-2 cells and diabetic rat kidneys against apoptosis induced by high glucose levels by targeting autophagy. As shown by our results, autophagy plays a potential role in nephropathy, which affects cell viability through the GLP-1 receptor.

## Materials and methods

### Cell culture

The human renal tubular epithelial cell line (HK-2) was purchased from the American Type Culture Collection (ATCC, Manassas, VA, USA) and was cultured in Dulbecco’s modified Eagle’s medium (DMEM) supplemented with 5.5 mM D-glucose [normal glucose (N)], 10% fetal bovine serum (FBS), epidermal growth factor, 100 U/ml penicillin, and 100 *μ*g/ml streptomycin (all from HyClone, Logan, UT, USA) in a 5% CO_2_ incubator at 37°C.

### 3-(4,5-Dimethylthiazol-2-yl)-5-(3-carboxymethoxyphenyl)-2-(4-sulfophenyl)-2H-tetrazolium (MTS) assay

The HK-2 cells were plated on 96-well plates at a density of 1.2×10^5^ cells/cm^2^ in medium containing either 5.5, 16.7, 25 or 40 mM glucose [high glucose (HG)] and incubated for up to 72 h. Liraglutide (LG) was administrated at various concentrations (1, 10 and 100 nM) or HG with LG with glucagon-like peptide-1 receptor (GLP-1R) antagonist {exendin-(9-39) [EX-(9-39)]; 1,000 nM}. At 24, 48 and 72 h, cell viability was assessed by the ability of metabolically active cells to reduce the tetrazolium salt to formazan compounds using MTS reagent (Promega, Madison, WI, USA). The absorbance of the samples was measured using a microplate reader at a 450-nm wavelength after 3 h of incubation with MTS solution (0.19 mg/ml). The results are expressed as the means ± standard error of the mean (SEM) and are representative of 3 independent experiments.

### Trypan blue exclusion assay

The cells were plated on 12-well plates at a density of 1.2×10^5^ cells/cm^2^ in medium containing either 5.5 or 40 mM glucose, collected and stained with trypan blue (Invitrogen, Carlsbad, CA, USA). The total number of total cells, as well as the number of trypan blue-stained cells were counted using a hemocytometer (Cat. no. 02-671-6; Hausser Scientific, Horsham, PA, USA).

### Western blot analysis

The cells were harvested and lysed in RIPA buffer (150 mM sodium chloride, 1.0% Triton X-100, 0.5% sodium deoxycholate, 0.1% sodium dodecyl sulfate, 50 mM Tris, pH 8.0) with protease and phosphatase inhibitors, and centrifuged at 12,000 rpm for 20 min at 4°C. Protein samples were then mixed with loading buffer and boiled at 95–100°C for 5 min. Total protein extracts were subjected to 12% SDS-PAGE. The separated proteins were transferred ono polyvinylidene fluoride membranes (Bio-Rad, Hercules, CA, USA) by electrotransfer. The blots were subsequently blocked with 5% (v/v) skimmed milk (Nacalai Tesque, Kyoto, Japan) and incubated with GLP-1R rabbit antibody (ab39072, 1:1,000; Abcam, Cambridge, MA, USA), LC3 rabbit antibody (12741S, 1:1,000) and Beclin1 rabbit antibody (3495S, 1:1,000) (both from Cell Signaling Technology, Danvers, MA, USA) for 12 h at 4°C, or with glyceraldehyde 3-phosphate dehydrogenase (GAPDH) antibody (G8795, 1:1,000; Sigma-Aldrich; St. Louis, MO, USA) for 1 h at room temperature. The membranes were incubated with horseradish peroxidase-linked, goat anti-rabbit (sc-2054) or anti-mouse IgG (sc-2055, 1:5,000; both from Santa Cruz Biotechnology, Inc., Santa Cruz, CA, USA) at room temperature for 2 h. The blots were then visualized using a western blotting detection system (ECL plus; GE Healthcare, Princeton, NJ, USA).

### Reverse transcription-quantitative (real-time) polymerase chain reaction (RT-qPCR)

Total RNA was extracted from each sample using the Total RNA kit I (Omega Bio-Tek, Norcross, GA, USA). cDNA was synthesized from the individual samples of 1 *μ*g of total RNA using the PrimeScript^®^ RT reagent kit (Takara Bio, Inc., Tokyo, Japan). Following the addition of each set of primers (final concentration, 0.4 *μ*mol/l) and template DNA to the master mix, quantitative (real-time) PCR was performed using a LightCycler (Roche Diagnostics, Tokyo, Japan) and SYBR Premix Ex Taq (Takara Bio, Inc.). The PCR protocol was as follows: initial denaturation (95°C for 30 sec) followed by 40 cycles of denaturation (95°C for 30 sec, 60°C for 30 sec and 72°C for 30 sec) and annealing and extension (72°C for 1 min). The specific oligonucleotide primers were designed by Takara Bio Inc., and the primer sequences were as follows: *GLP-1R* sense, TCAAGGTCAACGGCTTATTAGTGAA and antisense, CCCAAGTGATGCAAGCAGAG; *GAPDH* sense, GCAC CGTCAAGGCTGAGAAC and antisense, TGGTGAAGACGCCAGTGGA. To visualize gene expression, individual DNA fragments were electrophoresed on a 2% (w/v) agarose gel (Sigma-Aldrich) and treated with ethidium bromide. cDNA of the human pancreas (Takara Bio, Inc.) was used as a positive control.

### Electron microscopy

The HK-2 cells were plated in 0.01% poly-L-lysine (Sigma-Aldrich)-coated glass slides at a density of 1.5×10^4^ cells/slide (area, 1.8 cm^2^), cultured for 1 day, and finally treated for 72 h in medium containing either a 5.5 or 40 mM glucose concentration. The cells were fixed in 2.5% glutaraldehyde (Electron Microscopy Sciences, Hatfield, PA, USA) for 2 h and dissolved in 0.1 M phosphate buffer (PB; pH 7.4). The HK-2 cells were then post-fixed for 1 h in 1% osmium tetroxide in PB and then stained with 70% ethanol containing 1% uranyl acetate (Sigma-Aldrich). The HK-2 cells were then dehydrated in a graded alcohol series and embedded in epon (Sigma-Aldrich). Ultrathin sections (with silver to gray interference) were cut using a diamond knife (Diatome, Biel, Switzerland), mounted on Formvar-coated single-slot grids and then counterstained with 3% uranyl acetate and then with 0.2% lead citrate (Sigma-Aldrich). The sections were visualized under a Philips CM100 transmission electron microscope (Philips Electron Optics, Hillsboro, OR, USA).

### Animals

The animal care, handling and *in vivo* studies complied with the guidelines provided by the Animal Care Committee of the Fourth Military Medical University. Male Sprague-Dawley rats (4 weeks old) were divided into the following groups: i) non-diabetic group (n=10); ii) diabetic group (n=10); iii) diabetic group treated with liraglutide (n=10); and iv) diabetic group treated with liraglutide and the GLP-1R antagonist, exendin-(9-39) (synthesized by Sigma-Aldrich; n=10). At the age of 5 weeks, the mice in the diabetic groups were administered intravenous injections of streptozotocin (MP Biomedicals, Santa Ana, CA, USA) at 60 mg/kg body weight in citrate buffer (pH 4.5). Only the rats with blood glucose concentrations >16.7 mM at 3 and 7 days following the injection of streptozotocin were included in the diabetic groups. The non-diabetic groups were administered injections of citrate buffer alone.

The groups treated with liraglutide were administered liraglutide (Novo Nordisk, Copenhagen, Denmark) subcutaneously at the dose of 0.3 mg/kg/12 h for 5 weeks as previously described (33). Twice-daily dosing was used as the pharmacokinetic half-life of liraglutide is only approximately 4 h in rats. The mice in the group treated with liraglutide and the GLP-1R antagonist, exendin-(9-39), were subcutaneously administered liraglutide at the dose of 0.3 mg/kg/12 h and exendin-(9-39) at the dose of 25 nmol/kg/12 h for 5 weeks, beginning at 1 week after the streptozotocin or citrate buffer injections. The placebo groups were administered water alone using the same schedule as for the liraglutide treatment groups. All rats were allowed free access to standard food and tap water. All rats were euthanized at 5 weeks after the induction of diabetes in the diabetic groups, and the kidneys were weighed and fixed in 10% (v/v) formalin or frozen in liquid nitrogen.

### Assays of metabolic variables

Serum creatinine and blood urea nitrogen levels were measured using a BioMajesty JCA-BM12 analyzer (Hitachi, Tokyo, Japan). Body weight was monitored weekly from 4 weeks of age. Food intake was calculated as an average over a period of 3 days.

### Immunohistochemistry

Hematoxylin and eosin (H&E) and immunoperoxidase staining were performed as previously described (34). The kidneys were fixed in 10% formaldehyde, and embedded in paraffin. Paraffin sections were cut at 3 *μ*m and deparaffinized for staining. Briefly, for immunoperoxidase staining, the primary antibodies used were GLP-1R rabbit antibody (1:200; Abcam) and LC3 rabbit antibody (1:200; Cell Signaling Technology), and were applied for 12 h at 4°C. Secondary antibodies were biotin-labeled anti-rabbit IgG (Santa Cruz Biotechnology, Inc.), which were applied for 60 min at room temperature. The sections were counterstained with hematoxylin before being examined under a light microscope (Olympus, Tokyo, Japan).

### Statistical analysis

Data are presented as means ± SEM. Statistical analysis was assessed by one-way ANOVA followed by the least significant difference (LSD) t-test or Tamhane’s T2 for multiple comparisons. A P-value <0.05 was considered to indicate a statistically significant difference.

## Results

### Chronic exposure to high glucose concentrations decreases cell proliferation and induces apoptosis

DMEM containing 5.5 mM glucose has been used as a standard culture medium for HK-2 human renal tubular epithelial cells. In order to examine the cytotoxicity resulting from exposure to high glucose concentrations, cell viability was first measured by MTS assay, which is dependent on the metabolic activity of viable cells. The HK-2 cells were cultured in medium containing 5.5, 16.7, 25 or 40 mM glucose for 72 h. Cell viability significantly decreased in a glucose concentration-dependent manner (Fig. 1A). Of note, the HK-2 cells cultured in 40 mM glucose for 24 h at a density of 1.2×10^5^ cells/cm^2^ showed increased viability. After 72 h of culture in 40 mM glucose, however, there was a significant decrease in viability as compared to the cells incubated in medium with 5.5 mM glucose (Fig. 1B).

The decrease in MTS values observed with 40 mM glucose may be due to reduced proliferation or increased cell death. When cell death was assessed by the trypan blue exclusion assay, increased numbers of dead cells were observed at 72 h in the cells cultured with 40 mM glucose (Fig. 1C).

### Effects of liraglutide on HK-2 cell viability are mediated through GLP-1R

The HK-2 cells cultured in a high concentration of glucose for 72 h showed a significantly decreased cell viability. Liraglutide significantly enhanced cell viability in a dose-dependent manner. Additionally, the effects of liraglutide were significantly blocked by exendin-(9-39), a GLP-1R antagonist (Fig. 1D). The loss of viability that occurred in the cells at 72 h cultured in the presence of 5.5 or 40 mM glucose was associated with the activation of the common executioner caspase, caspase-3 at the protein level. Liraglutide downregulated caspase-3 expression, and exendin-(9-39) partly blocked this effect (Fig. 1E).

### Effect of liraglutide on GLP-1R expression in HK-2 cells

The HK-2 cells stimulated with a high concentration of glucose for 72 h showed significantly decreased levels of GLP-1R expression. Liraglutide significantly enhanced GLP-1R mRNA expression in a dose-dependent manner. Additionally, the effects of liraglutide were significantly blocked by exendin-(9-39). The protein expression of GLP-1R was altered in a similar manner (Fig. 2).

### Chronic exposure to high glucose concentrations alters cellular ultrastructure

Changes in the ultrastructure of HK-2 cells induced by high glucose were examined under a transmission electron microscope. No changes in cellular nuclei or membranes were observed in the HK-2 cells cultured in the presence of high glucose at 24 h (Fig. 3A). A large number of free-standing membrane structures and double-membrane vacuoles was observed in the cytoplasm after 48 h, which resembled pre-autophagosomal structures. Typical apoptotic changes, with chromatin condensation and nuclear fragmentation, were observed in the cells exposed to high glucose concentrations, and the accumulation of glycogen significantly increased after 48 h. Nuclear fragmentation and disappearance and the formation of a large number of vacuoles indicated cytoplasmic vacuolization (Fig. 3B).

### High glucose concentrations promote autophagy in HK-2 cells

The promotion of autophagy by exposure of the HK-2 cells to high glucose was confirmed by electron microscopy, showing an accumulation of autophagosomes (Fig. 3C and D, black arrows).

The HK-2 cells stimulated with a high concentration of glucose for 72 h exhibited an increased expression of the autophagic markers, LC3-II and Beclin1. Liraglutide significantly attenuated the increase in LC3-II and Beclin1 gene expression in a dose-dependent manner. Additionally, the effects of liraglutide were significantly blocked by the GLP-1R antagonist, exendin-(9-39) (Fig. 4).

### Metabolic variables

Body and organ weights are presented in Table I. The body weights of the rats in the diabetic groups at 5 weeks after the initiation of liraglutide treatment were significantly lower than those of the rats in the non-diabetic group. The weight of the kidneys in the diabetic rats, normalized to the body weight of the rats in the non-diabetic groups, was significantly higher than that of the rats in the non-diabetic group. No significant differences were observed among the different diabetic groups.

Food intake was significantly increased in the diabetic groups, but was decreased in the diabetic groups at 5 weeks after the initiation of liraglutide treatment compared with the diabetic groups not receiving liraglutide. Serum creatinine and blood urea nitrogen levels, which are markers of renal injury, progressively increased in the diabetic groups during the experiment. Liraglutide treatment significantly reduced serum creatinine levels, but not the blood urea nitrogen levels, compared to the values in the diabetic groups not treated with liraglutide at 5 weeks.

### Kidney morphology

The level of glomerular hypertrophy was significantly greater in the diabetic groups (Fig. 5B) than in the non-diabetic group (Fig. 5A). By contrast, liraglutide treatment inhibited glomerular hypertrophy in the rats in the diabetic group (Fig. 5C). The renal interstitium showed a significantly greater level of tubular hypertrophy and vacuolar degeneration in the diabetic groups than in the non-diabetic group. Liraglutide treatment improved this situation; however, its effects were blocked by exendin-(9-39) (Fig. 5D).

### High glucose concentrations promote autophagy in the kidneys of diabetic rats

Immunohistochemistry revealed that the levels of the autophagic marker, LC3-II, were significantly upregulated in the kidneys of the diabetic rats (Fig. 6B) compared to those of the rats in non-diabetic group (Fig. 6A). Similar to the results from the *in vitro* experiments, liraglutide significantly decreased the expression of LC3-II (Fig. 6C). Additionally, the effects of liraglutide were partially blocked by exendin-(9-39) (Fig. 6D).

## Discussion

The balance between the survival and death of renal tubular epithelial cells plays a crucial role in the pathogenesis of diabetic nephropathy. In the present study, we characterized high glucose-induced toxicity in renal tubular epithelial cells both *in vivo* and *in vitro* by means of several complementary assays, including cell viability, cell death assays and the assessment of the changes in the ultrastructure of HK-2 cells. The viability of renal tubular epithelial cells was markedly reduced and the number of dead cells, including those undergoing apoptosis, was significantly increased when the cells were treated for a prolonged period of time with high glucose concentrations.

The exposure of renal tubular epithelial cells to high glucose concentrations for 72 h *in vitro* resulted in the downregulation of GLP-1R expression. Treatment with liraglutide increased cell viability, while exendin-(9-39) reversed this effect. These results support the concept that the changes in cell viabiltiy are caused by the reversible effects of glucotoxicity. These findings are consistent with the hypothesis that the unresponsiveness to GLP-1 is partly due to the changes in its receptor, suggesting that liraglutide has a renoprotective function that at least partially involves an increase in GLP-1R expression.

Importantly, we demonstrated that the chronic exposure of renal tubular epithelial cells and the kidneys of nephritic rats to elevated glucose levels induced autophagy. Autophagy is a cellular pathway involved in protein and organelle degradation. It occurs at a basal level in the majority of cells and is important in cellular homeostasis and responses to human disease (35). Autophagy can be induced by a variety of conditions, including nutrient deprivation and growth-factor depletion and hypoxia. However, little is known of the mechanisms underlying glucose-induced autophagy in renal tubular epithelial cells. Electron microscopy, the gold standard for monitoring the formation of autophagosomes, was used to demonstrate an elevated autophagic activity in HK-2 cells, where abundant vacuolization, a widely known morphologic indicator for autophagic cell death, was observed after 72-h of incubation in mediujm containing a high glucose concentration.

The pro-autophagic effect of high glucose was associated with the expression of LC3-II. The formation of autophagosomes includes the formation of pre-autophagosomal membranes (phagophore or isolation membrane), which is initiated by a class III phosphoinositide 3-kinase (PI3K) complex that includes Beclin1, and the elongation of the isolation membrane, which is stimulated by two ubiquitin-like conjugation systems (Atg12-Atg5 and LC3-phosphatidyletha nolamine) (36,37). It has been demonstrated that the activation of Beclin1 is consistently associated with the induction of autophagy in cancer cells (38). LC3, which is associated with the control of autophagosome elongation, is the second essential ubiquitin-like protein. Cytosolic LC3-I is recruited to the membrane and interacts with phosphatidylethanolamine and is converted to LC3-II. Thus, LC3-II has been used as a marker of autophagy (39). In the present study, autophagy was induced by high glucose concentrations, as directly observed by the accumulation of autophagic vacuoles in the cytoplasm, as well as by the increase in the content of the autophagic markers, LC3-II and Beclin1. The prominent role of autophagy in the response of renal tubular epithelial cells to prolonged exposure to high glucose concentrations suggests that autophagy may be an effective therapeutic target for the treatment of diabetic nephropathy.

The addition of liraglutide to the high-glucose medium significantly increased the viability of the HK-2 cells that were exposed to high glucose alone. Liraglutide is a human incretin and GLP-1 analogue with high homology to the native hormone. The intestinal absorption of glucose stimulates its secretion, which increases insulin and decreases glucagon secretion (27). GLP-1 is associated with enhanced satiety, reduced food intake and weight loss. GLP-1 preserves β-cell morphology and function, and reduces cellular apoptosis (40). In the present study, we also found that liraglutide inhibited the apoptosis of HK-2 cells, which was accompanied by a significant decrease in autophagy, and that exendin-(9-39), a GLP-1R antagonist, blocked the cytoprotective effects of liraglutide. The same trends in cell viability, GLP-1R expression and autophagy suggested the potential connections in this pathological procedure of high glucose-induced toxicity in renal tubular epithelial cells.

The question of whether autophagy is the driver of cell death or a pro-survival process in response to certain stress conditions remains controversial. Although autophagy was initially described as a cytoprotective mechanism under conditions of nutrient deprivation, several lines of evidence have indicated a role for autophagy in promoting cell death (41–43), similar to the *in vivo* and *in vitro* results obseved in the present study. This indicates that liraglutide may also prevent injury in renal tubular epithelial cells by reducing the autophagy induced by exposure to high glucose and may be a promising therapeutic agent. Future studies are required to determine the precise mechanisms underlying the differential effects of liraglutatide on apoptosis and autophagy, and to optimize its cytoprotective effects.

## Figures and Tables

**Figure 1:** Chronic exposure to high levels of glucose (HG) decreases cell proliferation and induces apoptosis. (A) Cell viability was assessed by MTS assay in HK-2 cells cultured in DMEM containing 5.5, 16.7, 25 or 40 mM glucose for 72 h. ^*^P<0.05 and ^**^P<0.01 vs. 5.5 mM group. (B) Cell viability was assessed by MTS assay in HK-2 cells cultured in DMEM containing 5.5 [normal glucose (N) group] or 40 mM glucose [high glucose (HG) group] for 24, 48 or 72 h. ^*^P<0.05 vs. the corresponding sample from the N group at each time point. (C) Trypan blue (TB) exclusion assay was performed as a measurement of cell death. ^*^P<0.05 vs. normal glucose group at each time point. (D) Cell viability was assessed by MTS assay in HK-2 cells. Cells were cultured in medium containing 5.5 or 40 mM glucose (HG) or HG with liraglutide (LG) at various concentrations (1, 10 and 100 nM) or HG with LG with glucagon-like peptide-1 receptor (GLP- 1R) antagonist {exendin-(9-39) [EX-(9-39)]; 1,000 nM} for 72 h. ^*^P<0.001 vs. N; ^**^P<0.001 vs. HG; ^***^P<0.05 vs. HG + 100LG. Values are the means ± standard error of the mean (SEM). (E) Protein levels of the cleaved, active form of caspase-3 and glyceraldehyde 3-phosphate dehydrogenase (GAPDH) as an internal control were determined in HK-2 cells cultured in 5.5 or 40 mM glucose medium or HG with LG or HG with LG with GLP-1R antagonist EX-(9-39).

**Figure 2:** Effect of liraglutide (LG) on glucagon-like peptide-1 receptor (GLP-1R) expression in HK-2 cells. (A) Quantification of GLP-1R mRNA expression in HK-2 cells cultured in 5.5 [normal glucose (N)] or 40 mM glucose medium or high glucose (HG) with LG at various concentrations (1, 10 and 100 nM) or HG with LG with GLP-1R antagonist {exendin-(9-39) [EX-(9-39)] by RT-qPCR. Values [means ± standard error of the mean (SEM)] are presented as the fold change relative to glyceraldehyde 3-phosphate dehydrogenase (GAPDH). The experiment was repeated 3 times. ^*^P<0.001 vs. N; ^**^P<0.001 vs. HG; ^***^P<0.05 vs. HG; ^+^P<0.05 vs. HG + 100LG. (B) Protein levels of GLP-1R in HK-2 cells cultured in 5.5 or 40 mM glucose medium or HG with LG or HG with LG with GLP-1R antagonist EX-(9-39) by western blot analysis.

**Figure 3:** Changes in the ultrastructure of HK-2 cells induced by high glucose. (A) Controls. No changes in cellular nuclei or membranes were observed. (B) Changes associated with apoptosis following exposure to high glucose for 48 h. Chromatin condensation and nuclear fragmentation were observed. (C and D) Autophagosomes of cells treated with high glucose for 72 h. A large number of free-standing membrane structures and double-membrane vacuoles was observed (arrows).

**Figure 4:** Changes in the expression of autophagic markers in HK-2 cells induced by high glucose (HG). Protein levels of microtubule-associated protein 1 light chain 3 (LC3; LC3-I and LC3-II) and Beclin1 in HK-2 cells stimulated with 40 mM HG or HG with liraglutide (LG) or HG with LG with glucagon-like peptide-1 receptor (GLP-1R) antagonist [EX-(9-39); 1,000 nM].

**Figure 5:** Effect of liraglutide on kidney morphology. Kidney morphology: (A) Non-diabetic group. Normal glomerular. (B) Diabetic group; glomerular hypertrophy was observed significantly. (C) Diabetes + liraglutide group. Liraglutide treatment inhibited glomerular hypertrophy in the rats. (D) Diabetes + lira-glutide + exendin-(9-39) group. The effects of liraglutide were blocked by {exendin-(9-39) [EX-(9-39)]. Glomerular hypertrophy was observed. Magnification for all images, ×400.

**Figure 6:** Effect of liraglutide on LC3 expression in rat kidneys. Immunoperoxidase staining for LC3: (A) Non-diabetic group. LC3 expression was at a basal level. (B) Diabetic group. The LC3 expression increased significantly. (C) Diabetic + liraglutide group. The liraglutide could decrease the LC3 expression; (D) Diabetic + liraglutide + exendin-(9-39) group. The effects of liraglutide were blocked by {exendin-(9-39) [EX-(9-39)]. The LC3 expression increased slightly. Magnification for all images, ×400.

**Table I:** Metabolic variables of the 4 groups of rats at 5 weeks after the induction of diabetes.

Characteristics	N	DM	DM + LG	HG + LG + EX-(9-39)
Baseline				
Body weight (g)	127±4	131±5	128±3	129±3
Fasting blood glucose (mmol/l)	4.0±0.3	3.9±0.2	3.7±0.3	3.3±0.3
Four weeks after treatment				
Body weight (g)	345±11	221±13^a^	205±10^a^	209±18^a^
Food intake (g/day)	25.9±4.3	41.6±4.3^b^	28.5±4.6^c^	31.3±1.8
Fasting blood glucose (mmol/l)	4.8±0.4	26.7±4.2^a^	20.5±3.7^b^	20.3±4.3^b^
Relative kidney weight (g/kg)	6.1±0.2	12.1±0.4^a^	10.6±0.4^a^	10.8±0.5^a^
Blood urea nitrogen (mg/l)	9.0±1.2	20.9±2.3^b^	18.0±1.4^a^	16.6±2.2
Creatinine (mmol/l)	62.1±1.8	74.4±4.5^b^	63.9±3.1	67.3±2.9

Values are the means ± SEM; n=10 animals in the each group.

a P<0.001

b P<0.05 vs. non-diabetic group

c P<0.05 vs. diabetic group. SEM, standard error of the mean. N, normal glucose; DM, diabetic group; DM + LG, diabetic group treated with liraglutide; HG + LG + EX-(9-39), group treated with high glucose and liraglutide and exendin-39.
